# Assessment of the Pollution Load of Effluents Discharged from Higher Institutions in Ethiopia: The Case of Bahir Dar University Zenzelma Campus

**DOI:** 10.1155/2022/9021549

**Published:** 2022-06-29

**Authors:** Mekuanint Lewoyehu, Nibret Abeje, Solomon Addisu

**Affiliations:** ^1^Department of Chemistry, College of Science, Bahir Dar University, P.O. Box 79, Bahir Dar, Ethiopia; ^2^Department of Natural Resource Management, College of Agriculture and Environmental Science, Bahir Dar University, P.O. Box 79, Bahir Dar, Ethiopia

## Abstract

Waste from industries, universities, and other institutions makes water a scarce resource. Although higher institutions have an honorable and principled responsibility to the environment, most higher institutions are not performing sensibly; they discharge untreated solid and liquid wastes into the environment. The objective of this study was, thus, to assess the pollution load of effluents from Bahir Dar University Zenzelma campus, Ethiopia. Wastewater samples were collected and analyzed for physicochemical and biological qualities and heavy metal levels. The phosphate (17.2–216.17 mg/L), BOD_5_ (51–86 mg/L), ammonia (0.02–10.29 mg/L), turbidity (22–580 NTU), total suspended solids (230–1293.33 mg/L), electrical conductivity (241–1492.03 *μ*S/cm), and total hardness (111.67–490 mg/L) levels surpassed the wastewater discharge limit stated by WHO, environmental protection authority, Compulsory Ethiopian Standard, and Environmental Health and Safety guidelines and did not fit wastewater reuse standard for irrigation and livestock drinking. 100% of the samples were not fit for livestock drinking as the coliform bacterium count exceeded the threshold level. Copper (0.006–1.75 mg/L), lead (0.019–0.18 mg/L), and cadmium (0.007–0.196 mg/L) levels crossed the wastewater discharge limit and were not fit for irrigation and livestock drinking, while the level of manganese (nill–0.01 mg/L) was under the threshold limit. Values of the water quality parameters were higher on the downstream site than at the upstream site showing the pollution load of Zenzelma campus effluents on the local environment (*Ch'imbil* River); wastewater used for irrigation and livestock drinking is unsafe. Thus, it requires immediate waste management interventions and appropriate waste treatment before being released into the environment.

## 1. Introduction

### 1.1. Background of the Study

Freshwater could be very vital for the existence of all dwelling organisms. But it can be a supply of numerous transmission and chronic human illnesses if it contains bacteriological, chemical, and physical contaminants. Even though getting access to safe consuming water is vital for people, an expected 1.2 billion people around the area lack access to safe water, and near 2.5 billion are not supplied with good enough sanitation Khosla [1]. Arnell et al. [2] reported that 1.4 to 2.1 billion people dwelling in the world are in water-harassed situations. Research showed that approximately 3.1% of deaths (1.7 million) and 3.7% of incapacity-adjusted life years (DALYs) (54.2 million) worldwide are on account of dangerous water, terrible sanitation, and hygiene [3].

Consequently, the danger of waterborne illnesses is a critical public health concern in lots of developing international locations. With close to a billion people, a large number of dwellings in the developing world do not have access to safe and clean water [4]. The World Health Organization (WHO) stated that around 94% of the worldwide diarrheal burden and 10% of the total ailment burden are due to dangerous drinking water, insufficient sanitation, and terrible hygienic practices [5]. According to WHO [6], the quantity and severity of water pollutants issues may be defined as “every year, over five million people die from water-related illnesses, two million of the yearly deaths are of kids, in developing international locations, 80% of all illness is water-related, at any individual time, half of the population in developing international locations will be suffering from one or more of the primary water-related illnesses, 1/4 of kids born in developing international locations could have died earlier than the age of five, and the extraordinary majority of them could have been from a water-related ailment.”

In line with the reported literature [7], the quantity of water to be had in growing areas of Africa and the center of East and South Asia is decreasing sharply while the clean water is deteriorating hastily due to rapid urbanization, deforestation, land degradation, and so forth. In Africa, roughly 40% of the population do not currently have access to water supply and sanitation [8]. An examination performed in rural villages of Mohale Basin in Lesotho shows that drinking water was polluted through *Escherichia coli* (78% of unprotected water and 60% of protected water assets) and 59% of water samples include open defecation with bad control of hygiene exercise [9].

Regrettably, in developing countries like Ethiopia, water is constantly being infected and unsafe for human use because of the population boom, expansion in industries, and throwing away wastewater and chemical effluents into canals and different water resources. As stated by Das et al. [10] and Hossain et al. [11], solid waste production and its disposal have emerged as a dependent on top-notch situations in developing countries. In Ethiopia, over 60% of communicable diseases are caused by terrible environmental heath situations springing up from risky and insufficient water delivery and terrible hygienic and sanitation practices [12]. Approximately 80% of the rural and 20% of the city population have no access to safe water. Three-fourths of the health issues of children within the country are due to communicable diseases springing up from the environment pollution, especially water and sanitation. Forty-six percent of those under 5 years of mortality are because of diarrhea wherein water-related diseases occupy a high share. The Ministry of Health, Ethiopia, stated that 6000 children die every day from diarrhea and dehydration [12].

Studies conducted in Dire Dawa and Jimma, Ethiopia, discovered that 83.34–87.5% of water samples had been positive for bacterial signs [13]. Moreover, a research completed in North Gondar showed that springs (35.7%), wells (28.6%), and water lines (50%) had *Escherichia coli* [14].

Water pollutants happen due to the physical, chemical, bacteriological, and metallic contaminants released from industries, universities, and other institutions. As stated by Boyd [15], public health professionals typically agree that a few of the contaminants of drinking water and microbiological pathogens are the foremost, important danger exhibited through drinkable water. Microbial or chemical infection of water cannot be detected utilizing sense organs like sight, scent, or taste. The handiest way to realize if water is infected with microorganisms or chemical substances is to test it in the laboratory. Checking out all viable microbial pathogens in water remains a very high-priced and time-consuming procedure. Consequently, checking out the most unusual signs such as overall coliform, fecal coliforms, and *E. coli* microorganism is conducted to locate the first-rate of water pollution [16].

Heavy metals released into the ecosystem from geogenic and anthropogenic (mining, agrochemicals, and industrial effluents) activities are the alternative water pollution Devorak et al. [17]. Rehman et al. [18] said that the probably dangerous detail contaminations ultimately affect human beings through the ingestion of diseased water. Consequently, regular quantification of heavy metals is essential to perceive temporal versions and infection load in aquatic ecosystems [19].

In Bahir Dar town, water pollution due to liquid and solid waste disposal is a serious problem. Untreated solid and liquid wastes from the textile factory, tannery, and other paint factories in the town go off directly into the water bodies. Furthermore, two-thirds of all households in Bahir Dar town discharge wastewater into streets and flood water drainages which ultimately discharge into the Blue Nile River and other water sources [20]. Students' cafeterias, teaching and research laboratories, and clinics are among the sources of solid and liquid waste in colleges and universities. Although academic institutes have the honorable and principled responsibility to act responsibly towards the surroundings and be an example of waste administration, many academic institutions are not acting sensibly; they release huge untreated solid and liquid trashes into the environment. Therefore, studies on the pollution load of solid and liquid waste discharges from universities are very important to design methods for better administration of waste.

Although waste management packages in higher training establishments in industrialized international locations started greater than 20 years ago [21], in Ethiopian universities, there's little or no research has been carried out regarding the pollution load of wastes they discharge into the surroundings. Zenzelma campus in Bahir Dar University is located closer to the *Ch'imbil* River. A sizable amount of liquid waste has been generated on an everyday basis at the campus. But there is no incorporated waste management practice in place with the aid of the campus to prevent the potential pollution danger. The liquid wastes generated within the campus discharge into this river water which is used for exceptional purposes like livestock consuming and bathing with the aid of the downstream communities. In addition, the communities in this area grow vegetables and chat at the sides of this River with the usage of the wastewater.

This study, therefore, aimed to gauge the sound effects of Bahir Dar University Zenzelma campus sewages on the water quality of *Ch'imbil* River, Northwest Ethiopia.

### 1.2. Significance of the Study

This study helps to obtain the necessary data on the pollution load of wastes from the Zenzelma campus and to construct better handling and alternative waste management practices. It also helps to estimate the water quality status of *Ch'imbil* River that the dwellers use for different purposes.

### 1.3. Objectives

#### 1.3.1. General Objective

The overall objective of this study was to assess the effects of Zenzelma campus effluents on the water quality of Ch'imbil River.

#### 1.3.2. Specific Objectives

The aim of this study was specifically as follows:

- Analyzing the physical and chemical quality of *Ch'imbil River* water and wastewater released from the Zenzelma campus.
- Estimating the biological quality and the heavy metals levels of *Ch'imbil River* water and wastewater released from the Zenzelma campus.
- Comparing the quality of *Ch'imbil River* water with the national and international water quality standards.
- Assessing the impacts of Zenzelma campus effluents on the water quality of *Ch'imbil River*.

## 2. Materials and Methods

### 2.1. Description of the Study Area

Bahir Dar University is a university in the city of Bahir Dar, the capital of the Amhara Region in Ethiopia. Bahir Dar University comprises different campuses, the university main campus (Peda), the College of Business and Economics campus, the College of Agriculture and Environmental Science campus (Zenzelma), the Institute of Technology campus (“Poly”), the Institute of Law and Land Administration campus (Yibab), Ethiopian Institute of Textile and Fashion Technology (Selam), and College of Medicine and Health Science. This study was conducted at the Zenzelma campus (Figure 1). Even though any waste produced has the potential to poison the nearby environment as well as posing a public health threat, since the waste is not handled properly, no previous studies have been done on the pollution effects of effluents discharged from this campus. Therefore, this study aimed to assess the effects of Zenzelma campus effluents on the water quality of *Ch'imbil River*.

### 2.2. Study Period

In working institutions, people's activities vary with time. Because of this, the degree of solid and liquid trashes they produce also differ. Thus, time differences comprehensively influence the nature and volume of waste they release. Having this in mind, in this study, academic and administrative activities carries out in the campus were presumed. Therefore, samples were collected in the period between February and March 2022 during which the campus had a maximum number of students and staff populations.

### 2.3. Sampling Procedures

The sampling sites were identified and nominated as outlet_1_, outlet_2_, and outlet_3_ for the waste outlet canals; D_1_, D_2_, and D_3_ for the sampling points just after the waste flows from the main outlets; D_4_ for the downstream site, after the waste from the three outlets joined the *Ch'imbil River*; and U for reference sample taken from the upstream site (water from *Ch'imbil River* where waste from the campus does not enter). The description of the sampling sites with GPS coordinates is presented in Table 1. The sample from the upstream (before the effluent joined the river) was used as a reference.

All sampling materials were washed with detergent, rinsed with distilled water, soaked in 10% HNO_3_ for 24 hrs, rerinsed with deionized water, and finally air-dried [22]. Sample bottles were then labeled for the date of sampling and sampling site. Water samples taken from three different points of each site were mixed and eight composite water samples were collected: three samples from the waste outlets since the waste from the campus flow out in three different canals; three samples from the waste lines of each canal just after the waste moves some distance from the outlets; one sample from the most downstream site (after the effluents from the three outlets joined *Ch'imbil River*); and one reference sample from the upstream of *Ch'imbil River* (before the effluent joined *Ch'imbil River*).

pH, EC, turbidity, and TDS were measured in situ [23]. For laboratory analysis, samples were transported in an icebox and kept refrigerated at 4°C until analysis.

### 2.4. Equipment and Chemicals

The equipment, the chemicals, and the standard procedures of water quality analysis mentioned in the research conducted by Lewoyehu [24] were also used during the laboratory analysis of this study. pH meter, EC meter, hotplate, volumetric flasks, filter paper (Whatman no. 1), Dropper (0.5 to 1 mL), sample cells (1-inch square, 10 mL), turbidimeter (Nephelometric), sample bottle, hand lens vacuum pump, Palintest test tube, and photometer (Photometer 8000, England) are among the equipment used for the accomplishment of the research. An inductively coupled plasma optical emission spectrophotometer (PerkinElmer optima 8000 ICP-OES) with the operating conditions mentioned in Table 2 was used to determine the level of selected metals in the wastewater samples.

From the readings of the standard solutions (0.002–4.05 ppm), prepared from 100 ppm CPI International standard stock solution by serial dilution, adjusted *R*^2^ values in the range 0.9993–0.9998 were obtained (Figure 2).

HNO_3_ (69–72%), KCl (1 M), H_2_O_2_ (30%), H_2_SO_4_ (98%), HCl (37%), CaCl_2_ (anhydrous), standard tablets of phosphate, nitrate, sulfate, ammonia, alkalinity, hardness, buffer solutions (pH: 4.7 and 7.01), and laurel sulfate broth were used in the research. Distilled water was used throughout the research.

### 2.5. Analysis of Physicochemical and Biological Parameters

The physical, chemical, and biological water quality parameters, temperature, total suspended solids (TSS), turbidity, pH, electrical conductivity (EC), total hardness (TH), total dissolved solids (TDS), nitrate (NO_3_^−1^), phosphate (PO_4_^−3^), sulfate (SO_4_^−2^), biochemical oxygen demand (BOD_5_), ammonia (NH_3_), and thermotolerant count (TTC), were analyzed. The levels of copper, manganese, lead, and cadmium were determined.

Temperature, EC, TDS, turbidity, and pH of the water samples were measured in situ. The pH and EC meters were calibrated using buffer and KCl solutions. A 100 mL water sample was taken from the source and pH and EC values were directly measured. Turbidity was measured using a precalibrated turbidimeter (Nephelometric). 10 mL water sample was taken in cuvettes and readings were taken in Nephelometric turbidity units (NTU). The TSS and BOD_5_ of the water samples were analyzed using the reported methods [25, 26].

The chemical analyses for the determination of total hardness, ammonia, sulfate, phosphate, and nitrate were done following the manufacturer's instructions (Palintest Transmittance-display photometer). Aliquots of water sample were collected and filtered through 0.45 *μ*m pore size, 47 mm diameter filter paper. Filtered water samples were used as a blank for each site. The absorbance of the developed color complex was measured under a specified wavelength (640 nm for NH_3_, 570 nm for total hardness, and NO_3_^−1^). For the determination of NH_3_, SO_4_^−2^, PO_4_^−3^, and NO_3_^−1^, ammonia Salicylate Reagent, SulfaVer 4 sulfate reagent, PhosVer 3 phosphate reagents, NitriVer 5 nitrate reagent powder pillow, respectively, were added to a sample cell filled with 10 mL water and left for the reaction to take place. After the completion of the reaction, values were recorded from the photometer readings.

Bacteriological analyses of the water samples were done using the membrane filter technique [27]. The membrane filter apparatus sterilized with a ﬂame from a gas burner and swiped with alcohol-soaked cotton wool was used. 100 mL of water was filtered out, under vacuum, through membrane filter apparatus with a uniform pore diameter of 0.45 *μ*m. Bacteria retained on the surface of the grid filter paper were placed on a suitable prepared medium (lauryl sulfate broth in a sterile Petri dish) and incubated at a temperature of 44.5**°**C for 24 hours. The thermotolerant or fecal coliforms in the water samples grown into yellow colonies were directly counted.

### 2.6. Data Analysis

All water quality data were analyzed using Microsoft Excel and descriptive statistics. The obtained data are expressed as mean ± SD of triplicate measurements. The water quality parameters of the analyzed wastewater samples were compared to the national and international water quality standards. One-way ANOVA using SPSS version 22 followed by Tukey's post hoc multiple comparisons test was used.

## 3. Results and Discussion

### 3.1. Analysis of the Physicochemical Water Quality Parameters

The level of the physicochemical parameters of the analyzed wastewater samples is summarized in Table 3.

#### 3.1.1. Temperature

The temperature of the wastewater samples in this study varied from 23.93 ± 0.12 to 28.93 ± 0.12 °C (Table 3). The water sample from the upstream site was found to have the lowest temperature since this site had lower suspended solids and light could transmit easily. The maximum temperature of the wastewater samples of this study was greater than the one reported by Abrehet *et al.* [28] (19.8–21.7 °C) for the wastewater discharged from the Peda campus of Bahir Dar University. The measured values were however below the acceptable limit of WHO [16] and EPA [29] (<30 °C) (Figure 3). Except for the samples from outlet_1_ and outlet_3_, statistical differences were found in the temperature of the wastewater samples from different sites.

#### 3.1.2. Turbidity

Turbidity ranged from 22.00 NTU at U to 580.00 NTU at D_3_. ANOVA results showed significant differences except between the samples at outlet_1_ and outlet_3_. According to the environmental protection authority [29], the parametric value of turbidity for water leaving the treatment plant is 1.0 NTU. Based on the WHO recommendation, the maximum tolerable limit of turbidity for drinking water is 5 NTU. Comparing the turbidity results of this study with the given standards, the turbidity level of all samples was beyond the limits (Figure 4). The highest turbidity of the water sample from D_3_ was in line with the highest total suspended solids on this site as light could be highly scattered by the suspended organic matter and the turbidity value became high.

According to CPHEEO [30], water for landscaping, horticulture and agriculture, and vehicle exterior washing must have a turbidity of <2 NTU. According to US EPA, for wastewater to be reused, it should have turbidity of <2 NTU. Thus, none of the tested samples met these standards. Water with turbidities of ≤10 NTU is very clear water; water with turbidities of 50 NTU is cloudy; and water with turbidities of ≥100–500 is very cloudy to muddy. Thus, water from outlet_2_, D_2_, D_3_, and D_4_ is categorized as muddy and none of the studied samples are clear waters.

#### 3.1.3. Total Suspended Solids (TSS)

The TSS values of the tested water samples varied from 230.00 ± 0.00 to 1293.33 ± 2.89 mg/L. Significant variations were observed among the samples from dissimilar sites. According to the Environmental, Health, and Safety (EHS) guidelines, and provisional industrial effluent standards of Ethiopia, the TSS values for treated sanitary sewage discharges must be below 50 mg/L [31]. Based on this standard, all the analyzed wastewater samples surpassed the permissible limit (Figure 5). In India, the wastewater discharge standard for TSS is 100 mg/L for inland surface water, 600 mg/L for public sewers, and 200 mg/L for land irrigation. Even though the people grew vegetables and crops using the wastewater, the TSS of the wastewater from the campus was unfit for irrigation activity. Furthermore, water from the sampling site U was used for drinking; but the mean value of TSS was higher than the WHO admissible limit for drinking water. TSS results of the studied samples were higher than wastewater reuse standards stated by different countries: US EPA (<30 mg/L), EU directives (<10 mg/L) for all irrigation methods, Jordan (<15 mg/L), Israel (<10 mg/L), South Korea (<10 mg/L), Italy (<10 mg/L), Spain (<35 mg/L), Portugal (<60 mg/L) for vegetables consumed raw, and France (<15 mg/L) [32, 33]. In Ethiopian standards, the permissible TSS of wastewater quality for irrigation is 200 mg/L. Hence, all samples of this study surpassed the tolerable limit. TSS results of this study were higher than the TSS values (9–397.5 mg/L) obtained in the physicochemical characterization of effluents from beverage industries in Ethiopia as reported by Abrha and Chen [34]. Goraw and his coworkers reported lower TSS values (1–34 mg/L) when they studied anthropogenic fecal pollution impact in Bahir Dar, Ethiopia [35].

#### 3.1.4. Total Dissolved Solids (TDS)

The mean values of TDS varied from 188.50 (outlet_1_) to 838.37 mg/L (outlet_2_). Mean values showed a significant difference (*P*=0.001), with the value at outlet_2_ being higher than the other sites (Table 3). TDS should be in the range of 500–2000 mg/L to reuse wastewater for agricultural activities [36, 37]. The maximum TDS value obtained in this study was greater than the TDS value reported by Abrehet et al. [28] (608 mg/L) for Bahir Dar municipal canal effluents, and Dagne [38] (328 ppm) for urban wastewater in Addis Ababa.

#### 3.1.5. pH

APHA [39] mentioned that the pH of most natural waters is between 6.0 and 8.5. WHO has recommended an acceptable range of pH from 6.5 to 8.5. So, all pH results of this study were within the recommended range (Figure 6). The pH mean values were in the range of 6.73 for outlet_3_ and 8.10 for outlet_2_. The mean values did not show a significant difference for sites outlet_1_, D_1_, and U. As per EHS, wastewater to be discharged should have a pH in the range of 6 to 9. Accordingly, the pH values of all samples in this study were within the recommended range. Water with a pH of 8–10 is poor for livestock drinking as it may be infected with bacteria and may be a health hazard. Despite slight numerical variations, the pH results of this study were in agreement with the values reported by Abrehet et al. [28] (6.3–7.6) and Goraw et al. [35] (6.8–9).

#### 3.1.6. Electrical Conductivity (EC)

The mean values of conductivity ranged from 241.00 *μ*S/cm for outlet_3_ to 1492.03 *μ*S/cm for outlet_2_. The significant variations confirmed from the ANOVA results revealed that the number of dissolved ions responsible for the conductivity was not the same in the eight sites. Different countries have given different recommendations for the level of EC in wastewater to reuse the wastewater for agricultural activities: EC < 10 *μ*S/cm for uncooked vegetables (Spain), EC < 1000 *μ*S/cm for vegetables consumed raw (Portugal), and EC < 700 *μ*S/cm for food crops (South Korea). Accordingly, the wastewater discharged from the Zenzelma campus was not fit for the aforementioned irrigation purpose even though the local people grew vegetables and crops using the wastewater. Goshu and his coworkers studied the fecal contamination of Lake Tana and reported conductivity of 130 to 1200 *μ*S/cm [35]. Abrehet et al. [40] reported conductivity of 1050 *μ*S/cm for effluent water discharged from Bahir Dar Textile Factory.

#### 3.1.7. Total Alkalinity (TA)

The mean values of TA went from 145.00 mg/L for outlet_3_ to 1200 mg/L for outlet_2_. The mean values of TA varied significantly (*P*=0.001), with the value at outlet_2_ being significantly higher than other sites. According to WHO, TA for drinking water should be <75 mg/L. It was observed that water at sample site U was used for drinking in the local community even though the TA was beyond the permissible limit. The TA values in this study were higher than the values reported in the literature (180–269.80 mg/L) by Abrehet et al. [28] for Bahir Dar municipal canal effluents and (91–247 mg/L) by Abrehet et al. [40] for the wastewater effluents discharged from Bahir Dar Textile Factory, Ethiopia.

#### 3.1.8. Total Hardness (TH)

The mean of total hardness varied from 111.67 mg/L for outlet_3_ to 490 mg/L for D_3_. There was a significant difference among the sampling sites (*P*=0.001) with D_3_ being higher than other sites. According to the National Research Council [41] and National Academy of Sciences [42], in general, the hardness level of the analyzed samples for livestock drinking is categorized as moderately hard (outlet_3_) (61–120 mg/L), very hard (outlet_1_, outlet_2_, D_1_, U) (181–350 mg/L), and brackish (D_2_, D_3_, D_4_) (>350 mg/L). None of the sampling sites were safe even for livestock drinking. This can cause problems of low pressure and low flow watering systems in livestock due to the accumulation of insoluble calcium and magnesium carbonate deposits. According to WHO recommendation, drinking water should have a maximum TH of 100 mg/L. WHO also recommended a maximum TH of 100 mg/L for inland surface water. Therefore, none of the samples had an acceptable level of TH. TH values of 91–350 mg/L and 84–117 mg/L were reported by Abrehet et al. [28] and Abrehet et al. [40], respectively.

#### 3.1.9. Nitrate

The nitrate level of the studied samples ranged from 8 mg/L for U to 52.6 mg/L for outlet_2_. Nitrate concentration varied significantly (*P*=0.001), with the mean value at outlet_2_ being the highest. CPHEEO [30] recommended the maximum concentration of nitrate in treated wastewater for different uses to be 10 mg/L. Based on this standard, samples from outlet_2_, outlet_3_, D_1_, D_2_, D_3_, and D_4_ were above the recommended limit. Nitrate concentrations less than 400 mg/L in livestock drinking water may not be harmful to animal health. Therefore, the nitrate level of the samples was safe for livestock consumption; samples from outlet_2_ and outlet_3_ were safe for livestock with low nitrate feeds and a balanced diet. According to the CES and WHO, the tolerable limit of nitrate in human drinking water is 50 mg/L. Thus, the nitrate concentration of site U that the local people used for drinking was below the maximum limit. FAO recommended the nitrate limit in water for irrigation to be 45 mg/L. Thus, the nitrate level of water from outlet_2_ and outlet_3_ was not within the safe limit though the local community did irrigation activities using this wastewater. The industrial effluent standard of Ethiopia for nitrate is 50 mg/L [31]. Only the sample at outlet_2_ was out of this standard. Mohamed [43] reported a nitrate concentration of 3.8–70 mg/L for the wastewater discharged from the tannery, food, and textile industries in Addis Ababa. Even though the maximum nitrate concentration obtained in this study was lower than the maxim value reported by Mohamed [43], the value was very high as Zenzelma is an academic institution and is not expected to discharge toxic environmental pollutants to the environment.

#### 3.1.10. Phosphate

The phosphate level for the wastewater sample in this study was in the range of 17.2 mg/L for U to 216.17 mg/L for outlet_1_. The phosphate mean values of different sites were significantly different (*P*=0.001), with the mean value at outlet_1_ being the highest. According to the Environmental, Health, and Safety (EHS) guidelines, the phosphate discharge limit in wastewater is < 5 mg/L. Based on this limit, the phosphate level of wastewater samples from all sites was above the permissible limit (Figure 7). WHO recommended a phosphate concentration of 2 mg/L for industrial sewage and irrigation effluents. Phosphates should not exceed 0.05 mg/l in streams discharged into lakes or reservoirs, 0.25 mg/L in a lake or reservoir, and 0.1 mg/l in flowing waters [37]. The provisional industrial effluent standard of Ethiopia for phosphate is 0.7 mg/L. The allowable limit of phosphorus in drinking water is 5 mg/l as P_2_O_5_, equivalent to 2.2 mg/L P (SI no. 81 of 1988). This is well above natural levels and an annual median phosphate concentration of 0.03 mg/L P is cited as a limit to prevent eutrophication in surface waters [44]. So, the phosphate level of all samples in this study was higher than the maximum recommended level. FAO [45] recommended the phosphate concentration of water for irrigation to be 3 mg/L. Therefore, water from all sites of this study did not fit the recommended limit.

Abrha and Chen [34] reported phosphate concentrations in the range of 0.185–69.7 mg/L when they studied the physicochemical characteristics of effluents from the beverage industry in Addis Ababa, Ethiopia. Mohamed [43] reported a phosphate concentration of 1–31 mg/L when he studied wastewater discharged from the tannery, food, and textile industries in Addis Ababa. 0.2–4.5 mg/L of phosphate was reported by Abrehet et al. [28] for Bahir Dar municipal canal effluents. Therefore, the phosphate concentration of the wastewater released from this academic institution, the Zenzelma campus, was higher than the reported values. A very high concentration of phosphate (3927–4615 mg/L) was reported by Amare et al. [46] who researched the wastewater discharged from Mekelle University, Ethiopia.

#### 3.1.11. Sulfate

The sulfate of the analyzed wastewater samples varied from 7.33 mg/L at outlet_3_ to 100.67 mg/L at D_3_. Mean values of samples from different sites were significantly different (*P*=0.001) except for samples at outlet_1_ and U. The sulfate level of the studied samples was below the threshold level of sulfate (200 mg/L) to induce surface water pollution. The WHO allowable standard of sulfate concentration in drinking water is 250 mg/L; thus, the sulfate concentration of sample site U that the dweller communities used for drinking was within the safe limit. The maximum recommended sulfate concentration in water for calves and adults is 500 mg/L and 1000 mg/L, respectively. The sulfate concentration of the tested water samples was therefore below the maximum limit. The sulfate concentration of water for irrigation as stated by FAO [45] is 20 mg/L. Accordingly, water from outlet_2_, D_1_, D_2_, D_3_, and D_4_ was not fit for irrigation even though people in the area grew vegetables and crops on the sides of the canal using the wastewater. Abrehet et al. [28] reported a 0.52–47 mg/L sulfate concentration for Bahir Dar municipal canal effluents, while Amare et al. [46] reported a sulfate concentration of 1400–1619 mg/L for the wastewater discharged from Mekelle University.

#### 3.1.12. Ammonia

The ammonia level of the tested water samples ranged from 0.02 mg/L at U to 10.29 mg/L at outlet_3_. The industrial effluent standard of Ethiopia for NH_3_ is 4.5 mg/L. According to the environmental protection rules, the NH_3_ level in the discharge effluent should not exceed 5 mg/L. Thus, samples at outlet_1_, outlet_2_, outlet_3_, D_2_, and D_4_ surpassed the permissible limits (Figure 8). EPA recommended the parametric value of NH_3_ in drinking water to be 0.3 mg/L. Its permissible limit given by WHO and CES is 1.5 mg/L. Therefore, the NH_3_ level of site U that the local people used for drinking was below the maximum limit stated by WHO and CES. Mohamed [43] reported an NH_3_ level of 0.5 mg/L for effluents from the metal and nonmetal industries, and 300 mg/L for tannery effluents in Addis Ababa. Goraw et al. [35] reported 12 mg/L of NH_3_ in the study on fecal contamination impact on the water quality of Lake Tana, Ethiopia, while Abrha and Chen [34] reported a high level of ammonia (0.265–71 mg/L) for the beverage industries in Addis Ababa.

#### 3.1.13. Biochemical Oxygen Demand (BOD_5_)

The amount of BOD_5_ for all samples went from 51 mg/L (outlet_2_) to 86 mg/L (D_4_). ANOVA showed significant variation, with the value at D_4_ being the highest of all others. In water with a BOD_5_ level of above 5 mg/L, the water is considered somewhat polluted because there is usually organic matter present and bacteria are decomposing this waste. The higher the BOD_5_ value, the greater the amount of organic matter or food available for oxygen-consuming bacteria. BOD_5_ values increase when nutrient loads and accumulation of plant decaying matters in sampling points increase.

BOD_5_ results in this study were above the permissible levels given by the guideline ambient environment standards of Ethiopia for priority surface water pollutants concerning the protection of aquatic species (<5 mg/L), WHO (2.0–5.0 mg/L), EPA (<5 mg/L), and FAO (8 mg/L) (Figure 9). Mostly, unpolluted streams have a BOD_5_ that ranges from 1 to 8 mg/L [36]. According to EPA [44], the optimum BOD_5_ for stream water is ≤ 5 mg/L. In Ethiopia, the permitted limit of BOD_5_ for interpretation of greywater use for irrigation of vegetables likely to be eaten uncooked is 20 mg/L. Given that, the BOD_5_ level of all sampling sites crossed the permissible limit even though the local communities in the area used the wastewater to grow vegetables.

BOD_5_ values of the studied samples were higher than wastewater reuse standards stated by different countries: <10 mg/L for crops and <30 mg/L for processed food crops (US EPA), <10 mg/L for all irrigation methods (EU directive), <10 mg/L (Israel), <8 mg/L for food crops (South Korea), <20 mg/L (Italy), <60 mg/L for all crops except those consumed raw (France), and <10 mg/L (India) [32], and National Green Tribunal order, 2019.

Amare et al. [46] reported BOD_5_ values in the range of 11413–15493 mg/L; Abrha and Chen [34] reported BOD_5_ values in the range of 15–576 mg/L; Mohamed [43] reported BOD_5_ values of 15, 46, 249, 566, 913, and 1942 mg/L for wastes discharged from metal and nonmetal, textile, chemical, food, beverage, and tannery industries, respectively; Abrehet *et al.* [28, 40] reported BOD_5_ values of 4.3–40.3 mg/L and 17–42 mg/L for Bahir Dar Textile Factory effluents and Bahir Dar municipal canal effluents, respectively. This revealed that the BOD_5_ results of this study were higher than the values early reported, and hence there was a high pollution burden in this area.

### 3.2. Bacteriological (Thermotolerant Bacteria Count (TTC)) Analysis

To determine the bacteriological characteristics of the wastewater discharged from the Zenzelma campus, a TTC determination analysis was done. The TTC of the studied samples varied from 13 cfu/100 mL at outlet_2_ to 42 cfu/100 mL at D_4_ (Figure 10). There was a statistical difference among the sampling sites in which the maximum bacterial count was obtained at D_4_. The EPA, WHO, and ECS recommended a 0 cfu/100 mL for drinking water. From the result, one can see that the bacterial colony counts were all above the WHO and EPA guideline limit of 0 cfu/100 mL. Unexpectedly, sample point U located above the waste outlets of the campus was polluted with thermotolerant coliform (fecal coliform), even higher than the wastewater discharged through outlet_2_. This might have been due to feces and other wastes from anthropogenic sources (open-field defecation by humans and other animals). It is recommended that livestock drinking water contain less than 1 cfu (colony forming unit) per 100 mL for calves and 10 cfu per 100 mL for adult cattle. Based on the TTC result of this study, therefore, all sampling sites did not fit even the livestock drinking water quality. But it was evident that the local community used the wastewater for their livestock drinking. Although human drinking water must be free from bacteria (0 cfu/100 mL), sample site U with a TCC of 15 cfu/mL was used as a drinking water source for humans. This may be hazardous to human health as they can cause infectious diarrhea diseases transmitted by the fecal-oral route. Water temperature promotes bacterial growth as high temperature leads to degradation of organic matter which makes a suitable environment for bacterial growth. In this study, site D_4_ with higher temperature was found to have higher TCC than other sites.

### 3.3. Heavy Metal Content Analysis

The levels of Cu, Mn, Pb, and Cd in the analyzed wastewater samples are depicted in Table 4.

#### 3.3.1. Copper

Copper is essential for both humans and animals, but it can cause acute gastrointestinal effects if the amount is above the threshold limit. The level of copper in this study was in the range of 0.06 mg/L at outlet_3_ to 1.75 mg/L at D_3_ (Table 4). The copper level varied significantly among the sample sites, with the mean value at D_3_ being higher than the others. Water with a copper level of <0.5 mg/L is essential to animal health (cattle, sheep, and horses) (water quality chart for livestock, 2007, Agdex 400/716–2). However, greater than 0.5 mg/L may be fatal for sheep, and greater than 0.1 mg/L can oxidize flavor in cows' milk. Water with a copper level above 0.6 mg/L can result in liver damage in dairy cows, even though this is below the level considered toxic. In general, water with a copper level above 5 mg/L is toxic for the aforementioned animals. Given this standard, water at outlet_2_, D_2_, D_3_, and D_4_ was found not to be suitable for sheep and might cause liver damage in dairy cows. copper can be toxic to several plants at 0.1 to 1.0 mg/L in nutrient solutions. Due to this, the maximum tolerable concentration of copper in water for irrigation is 0.2 mg/L. Its allowed concentration in human drinking water is 2 mg/L. The concentration of copper in the studied samples was below the maximum permissible limit for human drinking water while only copper concentrations at outlet_1_ and outlet_3_ were below the maximum permissible limit of copper in irrigation water (Figure 11). Amare and his coworkers' reported a copper concentration in the range of 0.137–0143 mg/L for the wastewater discharged from Mekelle University [46].

#### 3.3.2. Manganese

The concentration of manganese in this study ranged from nil at outlet_3_ to 0.01 mg/L at D_3_. Mean values from different sites were significantly varied except for means for outlet_1_ and outlet_2_. In human drinking water, the maximum recommended concentration of manganese is 0.5 mg/L (WHO) and 0.2 mg/L (FAO). Its recommended limit for livestock drinking water is 0.05 mg/L, and 0.2 for irrigation water. Based on these standards, the level of manganese in the studied samples was below the permissible limit (Figure 12). A manganese concentration of 1.297–1.513 mg/L was obtained in the wastewater discharged from Mekelle University [46].

#### 3.3.3. Lead

The level of lead was in the range of 0.019 mg/L to 0.18 mg/L. Mean values of outlet_1_, D_1_, and D_2_ were not statistically different (*P* > 0.05). The maximum allowable level of lead is 0.01 mg/L for human drinking water, 0.1 mg/L for livestock drinking water, and 5 mg/L for irrigation water. lead can inhibit plant cell growth at very high concentrations (greater than the permissible limit). A high concentration of lead is toxic for animals and young animals tend to be more susceptible to lead poisoning than adults. Accordingly, the concentration of lead at all sites was above the recommended limit for human drinking water. While the lead concentration of outlet_2_ exceeded the recommended limit of lead for livestock drinking water, the values at all sites were below the threshold limit for irrigation water (5 mg/L) (Figure 13). Lead concentration obtained in this study was higher than the values reported by Amare et al. [46] (0.032–0.033 mg/L).

#### 3.3.4. Cadmium

Cadmium concentration ranged from 0.007 mg/L at U to 0.196 mg/L at outlet_2_. Mean values for different sites were statistically different, with the value at outlet_2_ being the highest of all others. The recommended maximum concentration of cadmium is 0.003 for human drinking water, 0.05 for livestock drinking water, and 0.01 for irrigation water. Thus, the cadmium concentration of all sample sites was above the recommended concentration of cadmium for human drinking water. Samples at outlet_1_ and U showed a cadmium concentration below the recommended maximum concentration of cadmium for livestock drinking water, while the remaining sample sites surpassed the allowable limit. The result showed that cadmium concentration at all sample sites except at U was above the recommended maximum concentration of cadmium for irrigation water though it was evident that the local people grew vegetables at the side of the campus using the wastewater (Figure 14). This was in agreement with the values reported by Amare et al. [46], where the concentrations of Co, Cd, Fe, and Mn were greater than the allowable limits.

## 4. Conclusions and Recommendations

### 4.1. Conclusion

The objective of this study was to estimate the environmental pollution effects of the waste discharged from the Zenzelma campus. The results indicated that the phosphate, BOD_5_, ammonia, turbidity, TSS, EC, total hardness, and to some extent nitrate levels surpassed the wastewater discharge limit stated by WHO, environmental protection authority (EPA), Compulsory Ethiopian Standard (CES), and Environmental, Health, and Safety (EHS) guidelines and did not fit wastewater reuse standard for irrigation and livestock drinking. 100% of the water samples were not fit for livestock drinking as the coliform bacterium (*thermotolerant indicator bacterium*) count exceeded the threshold level. Copper, lead, and cadmium levels crossed the wastewater discharge limit and were not fit for irrigation and livestock drinking. Values of water quality parameters were higher on the downstream site than those at the upstream site. This indicates the pollution burden of the Zenzelma campus effluents on the local environment (*Ch'imbil River*). Although wastewater from this campus did not fit the wastewater reuse standard for irrigation and is unsafe for livestock drinking, the local people used the wastewater for livestock drinking and grew vegetables at the sides of the campus. Thus, it requires immediate waste management interventions and appropriate waste treatment before being released into the environment.

### 4.2. Recommendations

Although, as an academic institution, the Zenzelma campus in Bahir Dar University has the moral and ethical obligation to act responsibly towards the environment, the campus discharges massive solid and liquid wastes into the environment without any pretreatment. The local people use this wastewater for irrigation and livestock drinking. This is hazardous for both humans and animals. Therefore, we strongly recommend that the campus has to build a waste treatment plant immediately and any waste should not be discharged before proper treatment.

In Ethiopia, wastewater reuse for irrigation activity is questionable. Therefore, regulatory standard charters should be developed and producers and consumers of toxic pollutants should act accordingly.

## Figures and Tables

**Figure 1:** Location map of the study site.

**Figure 2:** Calibration curves of the analyzed metals: manganese, cadmium, lead, and copper (A-D, resp.) with the concentration of 0.002, 0.004, 0.008, 0.016, 0.032, 0.05, 1.05, 2.05, 3.05, and 4.05.

**Figure 3:** Comparison of temperatures of wastewater from the Zenzelma campus and the WHO recommended maximum temperature limit in wastewater.

**Figure 4:** Comparison of the turbidity of wastewater from the Zenzelma campus and the maximum turbidity limit value for drinking water.

**Figure 5:** Comparison of TSS of the wastewater from the Zenzelma campus with the Ethiopian effluent discharge limit value and WHO standards.

**Figure 6:** Comparison between pH values of the effluents of the study sites and the Ethiopian wastewater effluent discharge limit value.

**Figure 7:** Comparison between phosphate level in wastewater from the Zenzelma campus and the ECS and WHO recommended phosphate discharge limit in wastewater.

**Figure 8:** Comparison between the NH_3_ level in wastewater from the Zenzelma campus and the ECS and WHO recommended NH_3_ discharge limit in industrial effluents.

**Figure 9:** Comparison between the BOD_5_ level in wastewater discharged from the Zenzelma campus and EPA recommended limit of BOD_5_ in wastewater to be reused for agricultural activity.

**Figure 10:** The level of thermotolerant bacteria in the analyzed wastewater samples.

**Figure 11:** Comparison of the copper concentration in wastewater discharged from the Zenzelma campus and the recommended limits of copper.

**Figure 12:** Comparison of the manganese concentration in wastewater discharged from the Zenzelma campus and the recommended limits of manganese.

**Figure 13:** Comparison of the lead concentration in wastewater discharged from the Zenzelma campus and the recommended limits of lead.

**Figure 14:** Comparison of the cadmium concentration in wastewater discharged from the Zenzelma campus and the recommended limits of cadmium.

**Table 1:** Description of the sampling sites.

Sampling site	Coordinates (UTM)	Descriptions
Outlet_1_	333325	First cannel through which waste from the campus (including waste from the clinic) moves out
	1285105	

Outlet_2_	332468	Second cannel through which waste from the campus (including waste from the animal farm) moves out
	1284908	

Outlet_3_	332296	Third cannel through which waste from the campus (including waste from dormitories and students' cafeteria) moves out
	1284816	

D_1_	332650	The sampling point after the waste flows some distance from outlet_1_
	1284924	

D_2_	332578	The sampling point after the waste flows some distance from outlet_2_
	1284837	

D_3_	332427	The sampling point after the waste flows some distance from outlet_2_
	1284718	

D_4_	332550	The downstream site, after which the waste from the three outlets joined the Ch'imbil River
	1284494	

U	332602	Upstream sampling point where reference samples were taken (water from *Ch'imbil River* where waste from the campus does not enter)
	1285237	

**Table 2:** ICP-OES operating conditions for each analyzed metal.

Parameter	Conditions	Metals	Wavelength (nm)
RF power (W)	1500 w	Cd	228.802
Plasma gas flow rate (L/min)	8	Pb	220.353
Auxiliary gas flow rate (L/min)	0.2	Cu	327.393
Nebulizer gas flow rate (L/min)	0.7	Mn	257.610
Plasma view	Axial		
Sample flow rate (L/min)	1		

**Table 3:** The physicochemical parameters of the studied water samples compared to the ECS and WHO guideline values.

SP	Temperature (°C)	Turbidity (NTU)	TSS (mg/L)	TDS (mg/L)	pH	EC (*µ*S/cm)	TA (mg/L)	TH (mg/L)	NO_3_^−^ (mg/L)	PO_4_^−3^ (mg/L)	SO_4_^−2^ (mg/L)	NH_3_ (mg/L)	BOD_5_ (mg/L)
Outlet_1_	24.50 ± 0.00^d^	38.67 ± 1.15^f^	480.33 ± 0.58^f^	288.00 ± 0.00^f^	7.03 ± .06^de^	329.00 ± 0.00^f^	268.0 ± 1.73^f^	185.0 ± 0.00^g^	9.10 ± 0.00^g^	216.17 ± 0.06^a^	18.00 ± 0.00^f^	9.88 ± 0.00^b^	66.0 ± 0.00^f^
Outlet_2_	22.90 ± 0.17^f^	184.00 ± 1.73^d^	710.33 ± 0.58^d^	838.37 ± 0.12^a^	8.10 ± 0.10^a^	1492.03 ± 0.06^a^	1200.0 ± 0.00^a^	350.0 ± 0.00^d^	52.60 ± 0.00^a^	208.90 ± 0.00^b^	47.33 ± 0.56^d^	4.84 ± 0.00^d^	51.0 ± 0.00^h^
Outlet_3_	24.30 ± 0.00^d^	36.00 ± 0.00^f^	420.00 ± 0.00^g^	188.50 ± 0.00^h^	6.73 ± 0.06^f^	241.00 ± 0.00^h^	145.0 ± 0.00^h^	111.67 ± 2.89^h^	46.00 ± 0.00^b^	30.80 ± 0.00^g^	7.33 ± 0.56^g^	10.29 ± 0.05^a^	73.07 ± 0.06^d^
D_1_	28.00 ± 0.00^b^	45.67 ± 0.58^e^	640.67 ± 1.15^e^	573.37 ± 0.12^e^	7.10 ± 0.00^d^	958.57 ± 0.12^e^	285.0 ± 0.00^e^	230.00 ± 0.00^e^	28.00 ± 0.00^e^	57.80 ± 0.00^f^	21.33 ± 0.56^e^	0.06 ± 0.00^f^	81.0 ± 0.00^b^
D_2_	26.07 ± 0.12^c^	290.33 ± 0.58^c^	810.33 ± 0.58^c^	605.37 ± 0.12^d^	7.83 ± 0.06^b^	1075.43 ± 0.31^b^	680.0 ± 0.00^b^	360.00 ± 0.00^c^	30.63 ± 0.06^d^	178.27 ± 0.12^d^	56.00 ± 0.00^c^	9.84 ± 0.05^b^	70.0 ± 0.00^e^
D_3_	27.80 ± 0.20^b^	580.00 ± 0.00^a^	1293.33 ± 2.89^a^	756.53 ± 0.15^c^	7.30 ± 0.10^c^	1068.33 ± 0.15^c^	360.0 ± 0.00^d^	490.00 ± 0.00^a^	30.90 ± 0.00^c^	190.20 ± 0.00^c^	100.67 ± 0.56^a^	2.42 ± 0.00^e^	78.0 ± 0.00^c^
D_4_	28.93 ± 0.12^a^	408.33 ± 1.53^b^	980.67 ± 1.15^b^	767.00 ± 0.00^b^	7.37 ± 0.06^c^	1007.90 ± 0.20^d^	459.33 ± 1.15^c^	410.00 ± 0.00^b^	25.60 ± 0.00^f^	146.27 ± 0.06^e^	76.00 ± 0.00^b^	8.79 ± 0.05^c^	86.26 ± 0.06^a^
U	23.93 ± 0.12^e^	22.00 ± 0.00^g^	230.00 ± 0.00^h^	201.00 ± 0.00^g^	6.87 ± 0.06^ef^	261.00 ± 0.00^g^	250.0 ± 0.00^g^	190.00 ± 0.00^f^	8.00 ± 0.00^h^	17.20 ± 0.00^h^	19.00 ± 0.00^f^	0.02 ± 0.00^f^	53.0 ± 0.00^g^
Average	25.80 ± 2.13	200.62 ± 40.69	695.71 ± 65.69	527.27 ± 51.79	7.29 ± 0.45	804.16 ± 90.88	459.92 ± 66.62	290.83 ± 25.47	28.85 ± 3.04	130.70 ± 16.09	43.21 ± 6.40	5.77 ± 0.87	69.71 ± 12.11
*P*-value	0.001	0.001	0.001	0.001	0.001	0.001	0.001	0.001	0.001	0.001	0.001	0.001	0.001
ECS	—	5	50	1000	6.5-8.5	1000	200	300	50	5	250	4.5	5
WHO	<30	5	20	500	6.5-8.5	300	75	100	50	2	250	1.5	5

TSS: total suspended solids; TA: total alkalinity; TH: total hardness, ECS: Ethiopian Compulsory Standard (National Standard). Values with different superscripts down the column are significantly different (*P* < 0.05).

**Table 4:** The studied heavy metal content of the analyzed wastewater samples.

SP	Cu (mg/L)	Mn (mg/L)	Pb (mg/L)	Cd (mg/L)
Outlet_1_	0.18 ± 0.00^g^	0.005 ± 0.00^c^	0.019 ± 0.00^f^	0.014 ± 0.00^g^
Outlet_2_	0.66 ± 0.00^d^	0.005 ± 0.00^c^	0.18 ± 0.00^a^	0.196 ± 0.00^a^
Outlet_3_	0.06 ± 0.00^h^	ND	0.024 ± 0.00^c^	0.081 ± 0.00^e^
D_1_	0.27 ± 0.01^f^	0.002 ± 0.00^f^	0.019 ± 0.00^f^	0.090 ± 0.00^c^
D_2_	1.3 ± 0.00^c^	0.004 ± 0.00^d^	0.019 ± 0.00^f^	0.16 ± 0.00^b^
D_3_	1.75 ± 0.00^a^	0.01 ± 0.00^a^	0.023 ± 0.00^d^	0.089 ± 0.00^d^
D_4_	1.5 ± 0.00^b^	0.006 ± 0.00^b^	0.02 ± 0.00^e^	0.08 ± 0.00^f^
U	0.32 ± 0.00^e^	0.003 ± 0.00^e^	0.026 ± 0.00^b^	0.007 ± 0.00^h^
Average	0.75 ± 0.13	0.004 ± 0.001	0.041 ± 0.011	0.090 ± 0.013
*P*-value	0.001	0.001	0.001	0.001
ECS	2	0.5	0.01	0.003
WHO	2	0.5	0.01	0.003

ECS: Ethiopian Compulsory Standard; ND: not detected.

## Data Availability

All datasets generated and/or analyzed during the current study are incorporated within this article.
